# Rhinosporidiosis of the Parotid Duct

This article has been retracted.

**DOI:** 10.1155/2014/131794

**Published:** 2014-01-28

**Authors:** Santosh Kumar Yadav, Suraksha Shrestha

**Affiliations:** ^1^Department of Oral and Maxillofacial Surgery, Chitwan Medical College Pvt. Ltd, P.O. Box 42, Bharatpur 10, Nepal; ^2^IAOMS Fellow Oral and Maxillofacial Oncology and Reconstructive Surgery, Department of Oral and Maxillofacial Surgery, Peking University School of Stomatology, 22 Zhongguancun South Avenue, Beijing 100081, China; ^3^Department of Prosthodontics, National Academy of Medical Sciences, Bir Hospital, P.O. Box 13606, Kathmandu, Nepal

## Abstract

Rhinosporidiosis is a benign chronic granulomatous infection caused by *Rhinosporidiosis seeberi* (*R*. *seeberi*). Rhinosporidiosis is endemic in South Asia, notably in Southern India and Sri Lanka. The common sites of involvement are the nose and nasopharynx followed by ocular tissue. Rhinosporidiosis is also known to involve many rare sites and may become disseminated to ocular in generalized form. Rhinosporidiosis of parotid duct is extremely rare. The case presented here is of 18-year-old male from the nonendemic zone of Nepal with a proliferative mass in the parotid duct. Although rhinosporidiosis was not taken into consideration in the clinical differential diagnosis, eventual histopathological diagnosis confirmed rhinosporidiosis. Thus clinicians should be flexible in the differential diagnosis of proliferative growth in the parotid duct, even in those cases which are from nonendemic areas.

## 1. Introduction

Rhinosporidiosis is a benign chronic granulomatous disease caused by *Rhinosporidium seeberi* (*R*. *seeberi*) [1]. It occurs sporadically and is known to be noncontagious. Although human rhinosporidiosis occurs universally with higher occurrence in parts of South Asia, it is endemic, especially in Southern India and Sri Lanka [2–4]. The most common site of infection in humans is the nose [1]. Other sites include the nasopharynx, larynx, oropharynx, conjunctiva, lacrimal sac, and genital mucosa. Intraorally, rhinosporidiosis is known to involve the lip, palate, and uvula, secondarily, by direct extension from nasal and nasopharyngeal lesions [1]. Primary involvement of the parotid duct is extremely rare.

We present a case of 18-year-old male from nonendemic zone of Nepal with proliferative mass in the parotid duct and recalcitrant to conventional management that subsequently showed the presence of *R*. *seeberi* on histopathologic analysis of the specimen.

## 2. Case Report

An 18-year-old male reported to the oral and maxillofacial department with complaints of swelling on left side of the face since 10 days, associated with a history of an increase in its size and also pain associated with swelling during meal time. No other associated symptoms were reported. There was no history of trauma in the recent past. Patient had history of consumption of unprocessed well water.

On clinical examination, patient was moderately built with no signs of parlor, jaundice, or lymphadenopathy. Systemic examination also did not reveal any abnormalities. The nose, nasopharynx, oropharynx, and eyes appeared normal. On local examination, there was a single, soft to firm consistency, discrete extraoral swelling on the left side of the cheek measuring about 4 × 3 cm, extending anteriorly to masseter muscle (Figures 1 and 2). Overlying skin was normal in color and texture with no local rise of temperature. There was tenderness felt on palpation with no fixity to underlying skin or structure. The mouth opening was restricted to 30 mm. Intraoral examination showed serious discharge from the mouth at the opening of inflamed Stensen's duct on milking the gland. Routine laboratory investigation revealed eosinophilia (eosinophils, 40%). The fine needle aspiration cytology (FNAC) showed presence of neutrophils and lymphocytes in the fluid with increased level of Amylase (9,02,651 U/L). Ultrasonography (USG) showed a cystic lesion in the subcutaneous plane of cheek of size 3 × 1.6 cm, with echogenic debris and internal septations, without demonstrable communication with Stensen's duct. Sialography of the left parotid gland showed contrast flow in the distal part of Stensen's duct with pooling of contrast in the area of the lesion (Figure 3). No demonstrable connection to the proximal part of the parotid gland was present which led to focal ductal dilation. A provisional diagnosis based on the clinical presentation and the investigations done diagnosed it as sialocele of the parotid duct. Surgical excision of the cystic lesion was planned under general anesthesia.

With the patient under nasoendotracheal intubation, owing to the position (subcutaneous plane) and size of lesion, incision of 2 cm was placed on the most prominent part of swelling (Figure 4). Intraoperatively, on skin dissection, a well encapsulated purplish, cystic mass was found in the cheek (Figure 5). The cystic lesion was identified as dilated segment of the parotid itself (Figure 6). The proximal and distal parts of the ducts were dissected further and were found to be in continuity with the cystic mass itself. The cystic mass was excised in toto, after clamping the distal and proximal ends of the parotid duct. Duct was cannulated with an infant feeding tube to maintain the continuity between the proximal and distal segments of the duct (Figure 7) and was secured with sutures.

The excised specimen was submitted for histopathologic examination. The hematoxylin-eosin-stained sections showed thin fibrocollagenous cystic wall lined by columnar to cuboidal to flattened cells. One of the parts of the specimen showed the presence of numerous, nonvital sporangia of *R*. *seeberi *(Figure 8). Histopathological examination confirmed the diagnosis of rhinosporidiosis of Stensen's duct with secondary infection and dilatation of the duct.

Expert opinion was sought to rule out possible involvement of the respiratory tract. Endoscopic sinuscopy was performed, which failed to reveal any nasopharyngeal rhinosporidiosis. Patient was treated with oral Dapsone under supervision of medical expert for 3 weeks. Postoperative period was uneventful and patient is on regular followup without any evidence of recurrence (Figure 9).

## 3. Discussion 

The pathogen *R*. *seeber*i was first discovered by Malbran in 1892 and later, cases in cattle were reported in India in 1894 [5]. It was first described by Seeber [6] in 1900 in the nasal region in his doctoral thesis of medicine [7].

Earlier classification of *R*. *seeberi* indicated that it was fungus, but Malbran, who discovered it, considered it as a sporozoan. On further research, this organism was considered to be a protozoan by Seeber [6] and phycomycete by Ashworth [8]. Finally, Herr et al. (1999) classified the organism *R*. *seeberi* as mesomycetozoea based on biological analysis of its ribosomal deoxyribonucleic acid [9].

Biochemical features such as synthetic pathways are not available for *R*. *seeberi*, whose biochemical and metabolic properties are, as with other mesomycetozoea, still unknown. Sexual stages, which are baseline in fungal taxonomy and nomenclature, are also unknown for *R*. *seeberi*.

Review of the literature shows frequency of the disease to be greater in South Asia, with the largest number of cases having been reported in Southern India and Sri Lanka [2–4]. This is the first case from the nonendemic zone of Nepal. Men are affected more than women (male : female ratio, 4 : 1) [1, 10]. Patients of all ages are affected, but the disease most frequently occurs in those aged between 20 and 35 years.

Common sites of involvement include the nose and upper respiratory tract [1]. As already mentioned, primary infection of the parotid duct is very uncommon [11, 12]. In our case the parotid was considered to be the primary site of inoculation of the organism because there were no other nasal or nasopharyngeal lesions.

The diagnosis of rhinosporidiosis is primarily made by observing the distinctive morphologic features of *R*. *seeberi* in affected tissue. Its life cycle begins in the tissue as a spore, and it passes through several stages of development from trophocyte to juvenile sporangium to mature forms with changes in thickness and lamination of walls. Nuclear condensation takes place to form endospores embedded in a mucoid matrix. Characteristically, special electron dense bodies of about 1 to 3 mm are seen in mature endospores. These endospores become extruded into the surrounding thick sporangial wall and eventually develop into trophocytes to perpetuate their life cycle [1, 4].

The most common mode of spread to host is by transepithelial infection or by autoinoculation. Infection with *R*. *seeberi* is most likely waterborne [3, 13, 14]. A high incidence has been observed in patients who dive and swim in stagnant water [12]. Individuals probably acquire the disease from water contaminated by diseased cattle. As our case patient had history of consumption of unprocessed well water. However, hematogenous spread and lymphatic spread are also reported [15]. They are thought to be responsible for dissemination of disease to anatomically unrelated sites.

Immunologic studies on rhinosporidiosis are remarkably scarce because of the inability to culture *R*. *seeberi* in vitro. Investigation on humoral immunity through dot-blot immunoassays showed significant levels of serum IgG, IgM, and IgA and salivary secretory IgA antibody in affected patients [16]. Cell mediated reactions in affected patients showed mixed cells in filtrate, with many plasma cells and fewer CD68^+^ macrophages, CD3^+^ T lymphocytes, and CD56/57^+^ natural killer cells; moreover, CD4^+^ T-helper cells are scarce. CD8^+^ suppressor/cytotoxic cells are numberous. These are indications that *R*. *seeberi *evades specific adaptive immunity through several mechanisms, which explains its enigmatic aspects such as chronicity, recurrence, and dissemination [9, 17].

Because the organism has not been isolated in culture, the histopathologic examination remains the gold standard for diagnosis [18]. The larger and thick walled sporangia of *R*. *seeberi* differentiate this lesion distinctly from the organism causing coccidioidomycosis [19]. The diagnosis can also be confirmed by a Giemsa-stained imprint smear of fine needle aspiration cytology [15].

The only drug which has been shown to have some rhinosporicidal effect is Dapsone, which arrests the maturation of sporangia and promotes fibrosis in the stroma, when used as an adjunct to surgery [20].

Treatment of choice is surgical resection [1, 11], as most recurrences occur due to spillage of endospores on adjacent mucosa. The patient was motivated to attend regular follow-up sessions and was reported to be disease free even after 3 years of followup.

The purpose of this report is to encourage clinicians to be flexible in the differential diagnosis of proliferative growth in the parotid duct, even in those from nonendemic areas.

## Figures and Tables

**Figure 1:** Preoperative (front view).

**Figure 2:** Preoperative (side view).

**Figure 3:** Sialography of the left parotid gland showing contrast flow in the distal part of Stensen's duct with pooling of contrast in the area of the lesion.

**Figure 4:** Incision marked over the most prominent part of swelling.

**Figure 5:** Intraoperative showing well encapsulated purplish cystic mass.

**Figure 6:** Showing dilated segment of parotid duct.

**Figure 7:** Showing duct cannulation with an infant feeding tube between the proximal and distal segments with normal salivary flow.

**Figure 8:** Hematoxylin-eosin-stained sections showing thin fibrocollagenous cystic wall lined by columnar to cuboidal to flattened cells and presence of numerous and nonvital sporangia of *R*. *seeberi*.

**Figure 9:** Postoperative.
